The article "Prognostic Factors of Combined Periodontal and Endodontic Lesions: A Retrospective Study" was published in 2022. Journal: Contrast Media Mol Imaging.

# Prognostic Factors of Combined Periodontal and Endodontic Lesions: A Retrospective Study

**DOI:** 10.1155/2022/5042097

**Published:** 2022-08-22

**Authors:** Jinhong Guo, Ying Li, Xuandong Lin, Xiaomei Yang, Wei Shi, Xiaoling Lu

**Affiliations:** ^1^College of Stomatology, Hospital of Stomatology, Guangxi Key Laboratory of Nanobody Research, Guangxi Nanobody Engineering Research Center, School of Basic Medical Sciences, Laboratory Animal Center, Guangxi Medical University, Nanning 530021, Guangxi, China; ^2^The Department of Stomatology, The Central Hospital Afilliated to Shandong First Medical University, Jinan 250013, China

## Abstract

**Objective:**

This study used a retrospective method to explore the relevant factors affecting the prognosis of periodontal-endodontic combined lesions.

**Methods:**

According to the changes of subjective feelings and clinical indicators of affected teeth, selected patients were divided into an effective group and an ineffective group. The natural conditions (age, gender, and smoking status) of the patients and various clinical indicators at the initial and follow-up visits were collected, including the periodontal clinical indicators of the whole mouth and the clinical indicators of the affected teeth. The full-mouth periodontal clinical indicators include periodontal probing depth (PD), clinical attachment loss (CAL), sulcus bleeding index (SBI), and simplified oral hygiene index (OHI.S); clinical indicators of affected teeth include PD, CAL, SBI, mobility (TM), clinical crown-to-root ratio (CR), periapical index (PAI), and number of root canals.

**Results:**

There were 74 cases of endodontic combined treatment, with a total of 86 teeth. There was no significant difference in age and gender ratio between the effective group and the ineffective group, and the proportion of smoking patients in the ineffective group was significantly higher than that in the effective group (*P* < 0.05). At the initial diagnosis, there was no significant difference in the clinical indicators of the whole mouth between the effective group and the ineffective group. After a combined endodontic treatment, the clinical indicators of the two groups were significantly improved (*P* < 0.01). There was no significant difference in other periodontal clinical indicators between the two groups.

**Conclusion:**

The prognosis of nonsurgical treatment of periodontal and periodontal combined lesions is mainly correlated to the patient's oral hygiene maintenance, as well as the loss of attachment, the degree of loosening, the clinical crown-to-root ratio, the periapical index, and the number of root canals.

## 1. Introduction

Periodontal and endodontic lesions (PEL) is mostly caused by bacterial infection that leads to the destruction of periodontal tissues and pulp tissues [1, 2]. It is not uncommon in clinical practice. Although the etiology and pathogenesis of periodontal disease and pulpal disease are different, there are mixed infections dominated by anaerobic bacteria in deep periodontal pockets, diseased pulp tissues, and periapical inflammatory tissues [3, 4]. In addition, there is also a linkage reaction between autoimmunity and inflammation in the pathogenesis of PEL [5, 6]. The infection and lesions of the two can spread and influence each other through special anatomical structures, resulting in the occurrence of combined lesions [7]. Because the PEL involves periodontal tissues, dental pulp, and periapical tissues, relating a variety of bacterial mixed infections, the anatomical structure of the communication between the two is special and complex, the clinical manifestations are diverse, and the treatment methods are complex [8, 9]. The diagnosis, treatment and prognostic evaluation of PEL are still difficult clinical problems.

The article "Prognostic Factors of Combined Periodontal and Endodontic Lesions: A Retrospective Study" was published in 2022. Journal: Contrast Media Mol Imaging.

The PEL involves both pulp tissues and periodontal tissues. Limited by the relative backwardness of diagnostic approaches, clinicians generally make a rough and preliminary judgment on the prognosis of PELs through their own practical experience at the current stage. The clinical manifestations of the PPD are diverse and complex; thus, the experience of clinicians alone is far from enough. Therefore, the determination of the prognosis of an individual patient must be based on the study of the prognosis of the disease group, and the research data of the large sample of the disease should be used as the premise, so as to make a scientific expectation of its prognosis [10].

In this study, a retrospective study method was used to collect the data and various clinical indicators of patients at the initial diagnosis and follow-up, to explore the relevant factors affecting the prognosis of PEL and to guide the prognosis judgment and treatment of PEL. The program has certain clinical significance.

## 2. Methods

### 2.1. Patients

72 cases of PEL were collected from December 2018 to December 2021, with a total of 86 teeth. The patient selection process is shown in Figure 1.

Patients including 42 males with 50 teeth and 32 females with 36 teeth. Patients were aged 24–66 years. The sample size of this experiment was determined by the sample size and power calculator, where the test level was two-sided *α* = 0.05, the test power was 0.8, and the confidence level was 95% as shown in Table 1.

### 2.2. Inclusion and Exclusion Criteria

The inclusion criteria for this study were as follows: (1) At the initial visit, the diagnosis was a case of PEL and the diagnosis was confirmed after treatment; (2) complete the relevant periodontal. The procedure of combined endodontic treatment: supragingival ultrasonic scaling at the initial visit, root canal treatment a week later, subgingival scaling and root planing 1 week after the completion of root canal treatment (two times), and periodontal maintenance treatment at the later stage; and (3) the disease records should be complete and should have various clinical indicators at the initial diagnosis, full-mouth curved body slices and root apical films of the affected teeth; various clinical indicators at 1, 3, and 6 months of follow-up after combined treatment, and 3 months after root canal treatment and 6-month-old periapical slices.

The article "Prognostic Factors of Combined Periodontal and Endodontic Lesions: A Retrospective Study" was published in 2022. Journal: Contrast Media Mol Imaging.

The exclusion criteria for this study were as follows: (1) abnormal tooth anatomy; (2) received periodontal treatment in the past 6 months before the initial visit; (3) take antibiotics or non-steroidal drugs in the past 3 months before the initial diagnosis; (4) related systemic diseases, such as hypertension, diabetes, and liver and kidney diseases; and (5) those who have incomplete records of relevant information in the chronicle of serious diseases.

### 2.3. Clinical Indicators

From the included patients, the clinical indicators of the patients were followed up for 1 month, 3 months and 6 months after endodontic treatment, including the periodontal clinical indicators of the whole mouth and the related indicators of the affected teeth. The periodontal clinical indicators of the whole mouth include PD, CAL, SBI and OHI-S; the periodontal indicators of the affected teeth include PD, CAL, SBI and TM; x-rays were taken 3 months and 6 months after the initial diagnosis and combined treatment, respectively The CR and PAI of the tooth were read from the X-ray film; the number of root canals of the tooth was mainly determined by root canal treatment（Figure 2）.

We probe to the gingival sulcus floor or cementum enamel boundary with a periodontal probe and record the mesial and middle of the labial (buccal) side of each tooth PD, CAL, and SBI at 6 sites of central, distal, and lingual (palatal) side mesial, central, and distal. Sulcus bleeding index (SBI): O = no bleeding on probing, healthy appearance of gingival margin and papilla; 1 = no bleeding on probing, but mild inflammation of gingival margin and papilla; 2 = point bleeding after probing; 3 = linear bleeding after probing, blood spilling in the gingival sulcus; 4 = bleeding after probing, blood spilling out of the gingival sulcus; 5 = bleeding or spontaneous bleeding after probing. Looseness (TM): According to the loosening direction of the teeth, the looseness in the buccal/labiolingual direction is grade I, the loosening in the buccal/labiolingual and mesiodistal directions is grade II, and the loosening in the buccal/labiolingual, mesiodistal and vertical directions is grade II degree III.

The article "Prognostic Factors of Combined Periodontal and Endodontic Lesions: A Retrospective Study" was published in 2022. Journal: Contrast Media Mol Imaging.

Simplified Oral Hygiene Index (OHI.S): The value is 0∼6, we check the labial (buccal) surface of 16, 1l, 26, 3l and the lingual surface of 36, 46, including the simplified soft scale index (DI.S) and simplified calculus index (CI-S). DI. S: 0 = no soft scale on the tooth surface; *l* = less than 1/3 of the tooth surface; 2 = between 1/3 and 2/3 of the tooth surface; 3 = more than 2/3 of the tooth surface. CI-S: 0 = no calculus above and below the gum; 1 = the calculus above the gingival occupies less than 1/3 of the tooth surface; 2 = the calculus above the gingival occupies between 1/3 and 2/3 of the tooth surface, or there is scattered subgingival calculus; 3 = supragingival calculus occupies more than 2/3 of the tooth surface, or there is continuous and thick subgingival calculus.

Clinical crown-to-root ratio (CR): The ratio of the lengths of the suprabone and infrabone teeth based on the apical radiograph of the affected tooth, with the horizontal line of the lowest point of the alveolar bone as the boundary.

Periapical index (PAI): According to the periapical film of the affected tooth, it is divided into grades 0–5, 0 = normal periapical bone density and no light-transmitting area; 1 = periapical light-transmitting area diameter of 0.5–1 mm; 2 = diameter of periapical light transmission area 1–2 mm; 3 = diameter of periapical light transmission area of 2–4 mm; 4 = diameter of periapical light transmission area of 4–8 mm; and 5 = periapical penetration The diameter of the light area is greater than 8 mm.

### 2.4. Grouping Criteria

Compared with the initial diagnosis, according to periodontal, the changes of patients' subjective feelings, and clinical indicators during the follow-up visit after combined endodontic treatment, the curative effect was divided into 3 groups (Table 2).

### 2.5. Statistical Methods

SPSS 21.0 software was used to analyze the natural conditions (age, gender, and smoking status) and various clinical indicators of the patients between the two groups. The *t* test was used to compare the differences in gender and smoking status of the patients between the two groups, the repeated measures analysis of variance was used to compare the differences in the clinical indicators of the full-mouth periodontium at different time points between the effective group and the ineffective group, and the independent samples *t* test was used to compare the differences of the patients between the two groups. There was no difference in age between the two groups.

The article "Prognostic Factors of Combined Periodontal and Endodontic Lesions: A Retrospective Study" was published in 2022. Journal: Contrast Media Mol Imaging.

## 3. Results

### 3.1. Comparison of Periodontal Clinical Indicators at Initial Diagnosis

In this study, PD, CAL, SBI, and TM of the teeth at the initial visit were selected as periodontal observation indicators. There was no significant difference in PD between the effective teeth and the invalid teeth. Observation indicators including CAL, SBI, and TM were higher in the invalid teeth than in the effective teeth, and the difference was statistically significant (*P* < 0.05, Figure 3).

### 3.2. Comparison of X-Ray Findings at Initial Diagnosis

CR and PAI reflect the damage of the alveolar bone around the affected teeth. The CR and PAI levels of the invalid teeth were higher than those of the valid teeth, and the difference was statistically significant (*P* < 0.05, Figure 4). The degree of alveolar bone destruction was more serious than that of the effective group.

### 3.3. Comparison of the Number of Root Canals between Effective Teeth and Invalid Teeth

The number of root canals in the affected tooth was determined by X-ray and root canal treatment. The average number of root canals of invalid teeth was more than that of valid teeth (*t* = 3.65, *P* < 0.05), and the difference was statistically significant.

### 3.4. Comparison of Clinical Indexes of Whole Mouth before and after Treatment of Effective Teeth and Invalid Teeth

All patients received a comprehensive periodontal system examination at the initial diagnosis, 3 months, and 6 months after the completion of the combined treatment, respectively. The comparison of the periodontal clinical indicators of the effective teeth and invalid teeth at the initial diagnosis and 3 months and 6 months after the treatment is shown in Table 3. In the patients included in this study, the severity of full-mouth periodontitis was moderate to severe, and there was no statistical significance in PD, CAL, SBI, and OHI-S between valid teeth and invalid teeth at the initial diagnosis. After combined treatment, the PD, CAL, SBI, and OHI-S were significantly improved (*P* < 0.01), but the OHI of invalid teeth. S was larger than the effective teeth, and the difference was statistically significant (*P* < 0.05). There was no statistical difference in other indicators (PD, CAL, and SBI) between the two groups.

## 4. Discussion

This study retrospectively included 74 patients with combined endodontic treatment with a total of 86 teeth. The patients were divided into an effective group and an ineffective group according to the subjective feelings of the affected teeth and the changes of clinical indicators. The natural status (age, gender, and smoking status) and various clinical indicators of the patients at the initial diagnosis and follow-up were collected, including the periodontal clinical indicators of the whole mouth and the clinical indicators of the affected teeth. Full-mouth periodontal clinical indicators include periodontal probing depth (PD), clinical attachment loss (CAL), sulcus bleeding index (SBI), and simplified oral hygiene index (OHI.S); clinical indicators of affected teeth include PD, CAL, SBI, range of motion (TM), clinical crown-to-root ratio (CR), periapical index (PAI), and number of root canals.

The article "Prognostic Factors of Combined Periodontal and Endodontic Lesions: A Retrospective Study" was published in 2022. Journal: Contrast Media Mol Imaging.

PD, CAL, and SBI are objective indicators reflecting the activity of periodontal inflammation and the damage and repair of periodontal tissue, an increase in these indicators represents the severity of PEL [11, 12], while OHI-S reflects the patient's oral hygiene maintenance and the increase of this index represents periodontal uncleanness [13, 14]. At the initial diagnosis, there was no significant difference in the periodontal clinical indicators between the effective group and the ineffective group. After combined treatment, PD, CAL, and SBI gradually decreased, indicating that the inflammation was alleviated and the periodontal tissue was recovering continuously. In the process of periodontal basic treatment, we carry out oral hygiene education for each patient, so that patients can master the method of oral hygiene maintenance. Therefore, OHI-S has been significantly improved after periodontal basic treatment. However, at 3 and 6 months after combined treatment, the simplified oral hygiene index of the ineffective group was higher than that of the effective group, indicating that the patients had poor oral hygiene maintenance, which may negatively affect the occurrence and development of PEL, accelerating the development of the disease. Therefore, it is necessary to continuously strengthen the oral hygiene guidance for patients received periodontal basic treatments to improve the therapeutic outcome.

The degree of periodontal tissue destruction of the affected tooth has a significant impact on the prognosis of PEL. PEL are mostly derived from moderate to severe periodontitis [15, 16]. Some scholars have proposed that severe periodontitis can lead to acute or chronic pulp inflammation, pulp congestion, and pulp necrosis [17]. The study found the hard tissue sections of teeth with severe periodontitis and found that bacteria were found in the dentin after root planing [17, 18]. After root planing, the cementum is lost and the dentin is exposed, so that the periodontal infection and the pulp are interconnected [19]. Therefore, conservative treatment should not be taken for the teeth with severe periodontitis [20]. In the results of this study, patients in the ineffective group were mostly treated with relatively conservative treatment plans, and the corresponding indicators such as PD, CAL, and SBI were also higher, suggesting that too conservative treatment plans may hinder the cure of the disease. Inflammation, which aids in the healing of periodontal tissue. Previous studies have shown that, for teeth with moderate-to-severe periodontitis with slow pulp vitality, the pulp of most of the teeth has undergone a certain degree of degeneration or necrosis [21, 22]. The infection in the periodontal pocket interacts with the inflammation in the root canal, which is beneficial to the control of periodontal inflammation, slowing down the development of lesions and promoting the healing of periodontal tissue, reducing the risk of periodontal surgery, thereby reducing the pain of patients [23, 24]. The greater the degree of periodontal tissue destruction, the worse the prognosis, and the conservative treatment should not be excessively conservative for the faithful teeth with moderate to severe periodontitis secondary to endodontic lesions, [25, 26]. In this study, patients treated conservatively had a poorer prognosis; PD, CAL, and other indicators are higher, which is consistent with the results of the above studies.

The article "Prognostic Factors of Combined Periodontal and Endodontic Lesions: A Retrospective Study" was published in 2022. Journal: Contrast Media Mol Imaging.

To sum up, the prognostic factors of PEL mainly include smoking and oral hygiene maintenance, loss of attachment, looseness, and clinical crown of the tooth. The root ratio, periapical index, and the number of root canals, as well as the doctor, can make a prognosis judgment on the affected tooth according to the specific situation of the patient, and make a targeted treatment plan considering the patient's wishes. Looking back at the development of medical care in recent years, the gradual deepening of PEL-related research studies, as well as the development and practicality of new drugs, has effectively improved the occurrence of oral diseases. In the field of medical practice, it is the focus of clinicians to make appropriate adjustments or updates to existing preventive methods, improve the patient's internal environment stability as much as possible, and reduce and eliminate adverse effects caused by PEL. It is also the focus of academic research and is an important direction.

## 5. Restrictions

The limitation of this study was as follows: we only included the teeth with clear periodontal and pulpal inflammation, blaming the difficulty in accurate diagnosis of periodontal and endodontic lesions. With the advancement of related technologies, more accurate diagnostic tools may be available in the future, which will benefit the accurate treatment of the symptoms of this disease, so that we can further include more manifestations of the affected teeth as samples for better correlation analyses. Although the subjective teeth without clear symptoms and clinical manifestations of pulpitis were not included, we still consider that the results of this paper have certain guiding significance for doctors to determine the prognosis of teeth with PEL.

The article "Prognostic Factors of Combined Periodontal and Endodontic Lesions: A Retrospective Study" was published in 2022. Journal: Contrast Media Mol Imaging.

## 6. Conclusion

The prognosis of nonsurgical treatment of periodontal and periodontal combined lesions is mainly related to the patient's oral hygiene maintenance, as well as the loss of attachment, the degree of loosening, the clinical crown-to-root ratio, the periapical index, and the number of root canals [6].

## Figures and Tables

**Figure 1:** Participant screening process.

**Figure 2:** (a) The photo of the patient at the time of operation; (b) the apical sheet; and (c) the X-ray film at the initial diagnosis.

**Figure 3:** Comparison of the periodontal index of the initial diagnosis between the effective teeth and invalid teeth. ^*∗*^: Statistical difference compared with the effective teeth (*P* < 0.05).

**Figure 4:** Comparison of X-ray findings between effective teeth and invalid teeth. ^*∗*^: Statistical difference compared with the CR (*P* < 0.05).

**Table 1:** General information for patients ($\bar{x}$ ± *s*).

Characteristics	General information (*n* = 74)
Gender (male/female)	42/32
Age (years)	47.54 ± 9.68
BMI	21.85 ± 3.21
Disease course (month)	7.23 ± 4.2

**Table 2:** Grouping criteria for patient response.

Degree	Characteristics
Cure	The patient has no symptoms, and the chewing function has improved. Clinical examination showed no gingival swelling, SBI <1, PD <3 mm, no increase in CAL, decrease in TM, no sinus or fistula on the buccal and lingual side, no percussion pain, and no shadow in the apical area on X-ray films. The alveolar bone density was normal

Improve	The patient had no symptoms, and the chewing function improved. Clinical examination showed mild inflammation of the affected teeth and gingiva, PD <4 mm, SBI <2, no increase in CAL, decrease in TM, no sinus or fistula on the buccal and lingual side, no percussion pain, and X-ray showed that PAl was decreased and less than or equal to 1

Invalid	The lesion continues to progress, the patient has conscious symptoms, and the teeth cannot drive to the normal chewing function. On clinical examination, the gums was red and swollen, PD >5 mm, increased CAL, SBI >3, TM, unchanged or enlargement of the sinus or fistula hole, percussion pain (+), X-ray showed the presence of shadows in the apical area and PAl

Among them, “cure” and “improve” are recorded as the effective group, and “invalid” is the invalid ineffective group.

The article "Prognostic Factors of Combined Periodontal and Endodontic Lesions: A Retrospective Study" was published in 2022. Journal: Contrast Media Mol Imaging.

**Table 3:** Comparison of periodontal clinical indicators between effective and ineffective teeth $\left(\bar{x}\pm s\right)$.

Characteristics	Clinical index	Effective tooth	Invalid tooth
Before treatment	PD	5.07 ± 1.25	4.64 ± 0.75
	CAL	3.25 ± 0.46	3.74 ± 0.24
	SBI	4.35 ± 0.95	4.18 ± 1.06
	OHI-S	3.15 ± 0.16	3.47 ± 0.32

3 months after treatment	PD	3.56 ± 1.01	3.74 ± 1.48
	CAL	2.67 ± 0.75	2.53 ± 1.01
	SBI	0.76 ± 0.12	1.25 ± 0.86
	OHI-S	1.25 ± 0.48	1.67 ± 0.47

6 months after treatment	PD	2.82 ± 1.08	3.21 ± 1.21
	CAL	1.64 ± 0.76	1.82 ± 1.02
	SBI	0.58 ± 0.32	0.92 ± 0.42
	OHI-S	0.72 ± 0.13	1.02 ± 0.72

## Data Availability

The data used to support the findings of the study are contained within the article or are available from the individual studies that were referenced throughout the text.
